The article "PTPN18 Stimulates the Development of Ovarian Cancer by Activating the PI3K/AKT Signaling" was retracted in 2023. Reasons: signs of a paper mill; suspected computer-generated content; unreliable results or conclusions; concerns about the data.

# PTPN18 Stimulates the Development of Ovarian Cancer by Activating the PI3K/AKT Signaling

**DOI:** 10.1155/2022/1091042

**Published:** 2022-03-11

**Authors:** Nan Mao, Hu Li, Hui Yang, Jianfen Su, Zhimin Liang, Guansheng He

**Affiliations:** ^1^Department of Pharmacy, Guangzhou Panyu Central Hospital, Guangzhou, China; ^2^Department of Gynecology, Guangzhou Panyu Central Hospital, Guangzhou, China; ^3^Department of Pharmacy, The Second Affiliated Hospital of Guangzhou Medical University, Guangzhou, China

## Abstract

**Objective:**

To illustrate the functions of protein tyrosine phosphatase nonreceptor type 18 (PTPN18) in the progression of ovarian cancer and the potential molecular mechanism.

**Methods:**

Differential PTPN18 expression in ovarian cancer samples was determined. Following PTPN18 knockdown, changes in proliferation and migration in ovarian cancer cells were detected. Nude mice with ovarian cancer were used to uncover the effects of PTPN18 on ovarian cancer growth in vivo.

**Results:**

PTPN18 was significantly upregulated in ovarian cancer samples and linked to pathological staging and metastasis rate. PTPN18 displayed prognostic and diagnostic potentials in ovarian cancer. Knockdown of PTPN18 and treatment of the PI3K inhibitor could inhibit proliferative and migratory abilities in ovarian cancer cells. Moreover, PTPN18 was capable of inactivating PI3K/AKT signaling. In vivo knockdown of PTPN18 suppressed ovarian cancer growth in nude mice.

**Conclusions:**

PTPN18 is upregulated in ovarian cancer, which stimulates the malignant development by activating PI3K/AKT signaling. The PTPN18 level is also associated with pathological staging and metastasis in ovarian cancer patients, which may be utilized as a hallmark predicting the malignant level.

## 1. Introduction

Ovarian cancer (OC) is one of the most common gynecological malignancies [1, 2]. Most patients are diagnosed as the advanced ovarian cancer or ovarian cancer accompanied by intraperitoneal implantation and metastasis, leading to a high mortality rate [1, 3]. Despite improvements achieved in surgical techniques and chemotherapy, the effective treatment rate of advanced OC is only 15–20% [4–6]. The Wnt, Notch, Hedgehog, and PI3K signaling are believed to influence the development of ovarian cancer [7–10]. At present, targeted therapy of ovarian cancer is well concerned. Clarifying ovarian cancer-associated signaling contributes to block the recurrence and metastasis, thus improving the clinical outcomes [11, 12].

Protein tyrosine phosphatase nonreceptor type 18 (PTPN18) is the first discovered specific tyrosine phosphatase of human epidermal growth factor receptor 2 (HER2), which is closely linked to tumor development [13, 14]. Protein tyrosine phosphatases influence cell growth and other cellular functions under external stimuli [13]. PTPN18 has a strict substrate specificity, and it can only dephosphorylate the phosphorylated tyrosine residues of HER2 [13, 15]. PTPN18 negatively regulates HER2 tyrosine kinase activity mainly through selectively dephosphorylating the tyrosine phosphorylation site of HER2, thereby effectively regulating cell function [13]. Previous evidence reported the expression of PTPN18 in kinds of tumor cell lines [13, 14]. In addition, it is able to inhibit the progression of chronic myeloid leukemia and to influence functions of hematopoietic stem cells [13, 14, 16].

As a vital pathway, the phosphatidylinositol 3-kinase/protein kinase B (PI3K/AKT) signaling is of significance in regulating cell activities [17, 18]. During tumor development, the PI3K/AKT signaling is overactivated, which is responsible for mediating malignant phenotypes of tumor cells [17–20]. Here, we explored the functions of PTPN18 and its potential mechanism in the malignant development of ovarian cancer.

## 2. Patients and Methods

### 2.1. Ovarian Cancer Patients Enrolled in the Study

Ovarian cancer tissues and paracancerous ones were collected from 44 patients without anticancer treatment. This study was approved by the Ethics Committee of Guangzhou Panyu Central Hospital (16GZ-EC403). Informed consent was also obtained from each subject before the study.

### 2.2. Cell Lines and Reagents

Six human-derived OC cell lines (SKOV3, OVCAR3, PEO1, A2780, 3AO, and CAOV3) and a human ovarian surface epithelial cell line (HOSEPiCs) were obtained from American Type Culture Collection (ATCC) (Manassas, VA, USA). Dulbecco modified Eagle medium (DMEM) supplemented with 10% fetal bovine serum (FBS) (Gibco, Rockville, MD, USA), 100 U/mL penicillin, and 100 *μ*g/mL streptomycin DMEM (Gibco, Rockville, MD) was used for cells culture in an incubator with 5% CO_2_ at 37°C.

### 2.3. Transfection

Cells with 30–40% confluence were transfected with transfection plasmids, GenePharma (Shanghai, China), via Lipofectamine 2000 reagent (Invitrogen company, Carlsbad, CA, USA).

### 2.4. Cell Counting Kit-8 (CCK-8) Assay

The cells were seeded in 96-well plates with 2×10^3^ cells in each well. The absorbance value of each sample at 490 nm was recorded using the Cell Counting Kit-8 (CCK-8) (Dojindo Laboratories, Kumamoto, Japan) at the specified time point to plot the survival curve.

### 2.5. Transwell Migration

700 *μ*L medium containing 10% FBS and 200 *μ*L suspension (5.0×10^5^/ml) was added to the upper and bottom of the transwell chamber (Millipore, Billerica, MA, USA), respectively. 48 h later, the fixed cells at the bottom were stained with crystal violet for 20 min. Finally, the number of migrating cells was calculated in 5 randomly selected regions in each sample.

### 2.6. qRT-PCR

RNA extracted with TRIzol reagent (Invitrogen, Carlsbad, CA, USA) was purified by the DNase I using PrimeScript RT reagent (TaKaRa, Otsu, Japan) and was reversely transcribed into cDNA. Quantitative real-time polymerase chain reaction (QRT-PCR) was performed on the obtained cDNA using SYBR^®^ Premix Ex Taq™ (TaKaRa, Otsu, Japan). The 2^−ΔΔC^ method was used for the analysis of the relative level of PTPN18 normalized to glyceraldehyde-3-phosphate dehydrogenase (GAPDH). PTPN18: forward: 5′-TTAATGGCAACTTCATCCG-3′, reverse: 5′-TCACCTTGACCCCAAACTC-3'; GAPDH: forward: 5′-TGACTTCAACAGCGACACCCA-3′, reverse: 5′-CACCCTGTTGCTGTAGCCAAA-3'.

### 2.7. Western Blotting

Cells were lysed to separate proteins. Protein was loaded on polyvinylidene fluoride (PVDF) membranes (Millipore, Billerica, MA, USA). Then, membranes were blocked in 5% skim milk for 2 hours. After being incubated with primary and secondary antibodies, the band exposure and analysis were performed.

### 2.8. Nude Mice Tumorigenicity Assay

The animal ethics and use committee approved the experimental procedures for the in vivo xenograft model of ovarian cancer in nude mice. Ten male nude mice were randomly divided into two groups (*n* = 5) and were injected subcutaneously with A2780 cells transfected with sh-NC and sh-PTPN18#1, respectively. Tumor size was recorded weekly. Mice were sacrificed after 6 weeks to collect tumor tissue. Ovarian cancer tissue sections from nude mice were blocked and incubated with anti-PTPN18.

### 2.9. Statistical Analyses

SPSS 19.0 software (IBM, Armonk, NY, USA) was used for data analyses. Comparison between multiple groups was done using the one-way ANOVA test followed by the post hoc test (least significant difference) (with 95% confidence interval). Percentage (%) was used to express the enumeration data, and the chi-square test was used for data analysis. Kaplan–Meier and ROC curves were depicted for analyzing the prognostic and diagnostic potentials of PTPN18 in ovarian cancer, respectively. *P* < 0.05 was considered as statistically significant.

## 3. Results

### 3.1. Upregulation of PTPN18 in Ovarian Cancer Samples

We found higher level of PTPN18 in OC tissues than paracancerous tissues (Figure 1(a)). Identically, PTPN18 was highly expressed in OC cell lines (Figure 1(b)).

The median level of PTPN18 was calculated in 44 included OC tissues. Subsequently, patients were divided into the high PTPN18 group or low PTPN18 expression group, respectively. It showed that PTPN18 level was positively linked to pathological staging, lymphatic metastasis, and distant metastasis in OC patients (Table 1). In addition, survival analysis demonstrated that PTPN18 was a risk factor of prognosis in OC (Figure 1(c)). ROC curves confirmed the diagnostic potential of PTPN18 in ovarian cancer (Figure 1(d)).

### 3.2. Knockdown of PTPN18 Attenuated Proliferation and Migration in OC

Transfection of either sh-PTPN18#1 or sh-PTPN18#2 could significantly decrease PTPN18 in A2780 and CAOV3 cells (Figure 1(e)). Knockdown of PTPN18 decreased viability in ovarian cancer cells (Figure 2(a)). Moreover, the number of migratory cells was lower in A2780 and CAOV3 cells with sh-PTPN18#1 or sh-PTPN18#2 than those of controls (Figure 2(b)).

### 3.3. Knockdown of PTPN18 Inactivated PI3K/AKT Signaling in Ovarian Cancer

Transfection with sh-PTPN18#1 or sh-PTPN18#2 decreased p-PI3K, p-AKT, and p-mTOR in A2780 and CAOV3 cells (Figure 3(a)). To further explore the interaction between PTPN18 and PI3K/AKT pathways, LY294002 (inhibitor of PI3K) was applied. LY294002 induction decreased protein level of PTPN18 in ovarian cancer cells (Figure 3(b)). Viability and migratory cell number in A2780 and CAOV3 cells were also reduced following LY294002 treatment (Figures 3(c), 3(d)).

### 3.4. Knockdown of PTPN18 Inhibited Tumorigenesis of Ovarian Cancer

A2780 cells with sh-NC or sh-PTPN18#1 were administrated into the left armpit of nude mice. Apparently, tumor volume was significantly smaller in OC tissues of mice with PTPN18 knockdown (*P* < 0.05) (Figure 4(a)). As expected, knockdown of PTPN18 markedly decreased the weight of harvested ovarian cancer (*P* < 0.001) (Figure 4(b)). Both Western blot and IHC results showed significantly lower level of PTPN18 in ovarian cancer tissues harvested from mice administrated with sh-PTPN18#1 than those of controls (*P* < 0.001) (Figures 4(c), 4(d)).

## 4. Discussion

Ovarian cancer is featured by high malignant level, fast growth, and high metastasis rate. Metastasis and recurrence are the two major events resulting in poor prognosis in ovarian cancer patients. In addition, endocrine therapy, TCM therapy, target drugs, and immunity treatment are also beneficial to ovarian cancer patients. Early discovery and diagnosis of cancer are of great significance. It is urgent to seek for effective hallmarks and therapeutic targets of ovarian cancer.

PTPN18 has been identified to regulate tumor cell behaviors. Our findings uncovered that highly expressed PTPN18 was associated with pathological staging and metastasis in ovarian cancer patients. Silence of PTPN18 remarkably suppressed proliferation and migration in OC cells. Moreover, in vivo knockdown of PTPN18 inhibited tumorigenesis in nude mice bearing ovarian cancer, manifesting as smaller tumor size and lower tumor weight than those of controls. It is demonstrated that PTPN18 was an oncogene in ovarian cancer.

Abnormally activated PI3K/AKT signaling is capable of stimulating tumor cell growth and metastasis [17, 18]. PI3K can specifically phosphorylate the 3-hydroxy group in inositol phosphate ring [17, 19]. Akt, also known as PKB, is the downstream target of PI3K [18–20]. Knockdown of PTPN18 decreased p-mTOR p-PI3K and p-AKT in OC cells. Application of LY294002, the PI3K/AKT inhibitor, achieved the same results as PTPN18 knockdown in ovarian cancer cells. Collectively, PTPN18 contributed to ovarian cancer deterioration by activating PI3K/AKT signaling. There are very obvious deficiencies in this study. For example, we simply tested the role of PTPN18 in several ovarian cancer cell lines. The effects of knockdown or overexpression of PTPN18 in mice models should be further explored. Additionally, the sample of the OC patients was small, which seriously weakened the evidence level of our conclusions. In the future, we plan to enlarge the sample size and also to further perform the in vivo experiments, thus to deeply investigate the biofunctions PTPN18 in OC and to elucidate the potential underlying molecular mechanism in the process.

## 5. Conclusions

PTPN18 is upregulated in ovarian cancer, which stimulates the malignant development by activating PI3K/AKT signaling. The PTPN18 level is also associated with pathological staging and metastasis in ovarian cancer patients, which may be utilized as a hallmark predicting the malignant level.

## Figures and Tables

**Figure 1:** Upregulation of PTPN18 in ovarian cancer samples. (a) Differential expression of PTPN18 in OC tissues and paracancerous ones. (b) PTPN18 level in ovarian cancer cell lines. (c) Overall survival in ovarian cancer patients based on their PTPN18 level. (d) ROC curves showing specificity and sensitivity in diagnostic potential of PTPN18 in ovarian cancer. (e) Transfection efficacy of sh-PTPN18#1 and sh-PTPN18#2 in A2780 and CAOV3 cells. Data are expressed as mean ± SD. ^∗∗^*P* < 0.05, ^∗∗^*P* < 0.01, ^∗∗∗^*P* < 0.001.

**Figure 2:** PTPN18 knockdown inhibited proliferation and migration of OC. (a) Viability in A2780 and CAOV3 cells transfected with sh-NC, sh-PTPN18#1, or sh-PTPN18#2, respectively. (b) Migration in A2780 and CAOV3 cells with sh-PTPN18#1, sh-PTPN18#2, or sh-NC, respectively (magnification: 40×). ^*∗*^*P* < 0.05.

**Figure 3:** Knockdown of PTPN18 inactivated PI3K/AKT signaling in ovarian cancer. (a) Protein levels of p-AKT, AKT, p-mTOR, p-PI3K, PI3K, and mTOR in A2780 and CAOV3 cells transfected with sh-NC, sh-PTPN18#1, or sh-PTPN18#2, respectively. (b) Protein level of PTPN18 in A2780 and CAOV3 cells induced with LY294002. (c) Viability in A2780 and CAOV3 cells induced with LY294002. (d) Migration in A2780 and CAOV3 cells induced with LY294002. ^∗^*P* < 0.05, ^∗∗^*P* < 0.01.

**Figure 4:** PTPN18 knockdown inhibited tumorigenesis of ovarian cancer. (a) Tumor volume that was weekly recorded in nude mice administrated with A2780 cells transfected with sh-NC or sh-PTPN18#1. (b) Tumor weight in nude mice administrated with A2780 cells transfected with sh-NC or sh-PTPN18#1. (c) Protein level of PTPN18 in ovarian cancer tissues collected from nude mice administrated with A2780 cells transfected with sh-NC or sh-PTPN18#1. (d) Positive level of PTPN18 in ovarian cancer tissues collected from nude mice administrated with A2780 cells transfected with sh-NC or sh-PTPN18#1. ^∗^*P* < 0.05, ^∗∗^*P* < 0.01.

**Table 1:** Clinicopathologic characteristics of the enrolled patients with ovarian cancer in low and high PTPN18 groups.

Indexes	*N*	PTPN18		*P*
		Low (*n* = 24)	High (*n* = 20)	
Age (y)				0.956
<60	20	11	9	
≥60	24	13	11	
T staging				0.047
T1/T2	26	17	9	
T3/T4	18	7	11	
Lymph node metastasis				0.040
No	25	17	8	
Yes	19	7	12	
Distance metastasis				0.019
No	28	19	9	
Yes	16	5	11	

## Data Availability

The datasets used and analyzed during the current study are available from the corresponding author upon request.
